# Observational study: daily treatment with a new compound “tradamixina” plus serenoa repens for two months improved the lower urinary tract symptoms

**DOI:** 10.1186/1471-2482-12-S1-S22

**Published:** 2012-11-15

**Authors:** Fabrizio Iacono, Domenico Prezioso, Ester Illiano, Antonio Ruffo, Giuseppe Romeo, Bruno Amato

**Affiliations:** 1 Department of Urology – University Federico II of Naples, Via S. Pansini, 5 – 80131 Naples – Italy; 2 Department of General, Geriatric, Oncologic Surgery and Advanced Technologies,-University “Federico II” of Naples. Via Pansini, 5 - 80131 – Naples, Italy

## Abstract

**Background:**

Lower urinary tract symptoms (LUTS) are associated with great emotional costs to individuals and substantial economic costs to society. This study seeks to evaluate the effect of a new natural compound “Tradamixina plus Serenoa Repens” in order to improve lower urinary tract symptoms.

**Methods:**

100 patients (≥45years) who had had LUTS/BPH for >6 mo at screening and with IPSS -The international Prostate symptom scores- ≥13 and maximum urinary flow rate (Qmax) ≥4 to ≤15 ml/s. were recruited. The compound “Tradamixina plus Serenoa Repens” (80 mg of Alga Ecklonia Bicyclis, 100 mg of Tribulus Terrestris and 100 mg of D-Glucosamine and N-Acetyl-D-Glucosamine plus 320 mg of Serenoa Repens) was administered daily for 2 months. At visit and after 60 days of treatment patients were evaluated by means of detailed medical urological history, clinical examination, laboratory investigations (total PSA), and instrumental examination like urolfowmetry. Efficacy measures included IPSS-International Prostate Sympto, BPH Impact Index (BII), Quality-of-Life (QoL) Index. Measures were assessed at baseline and end point (12 wk or end of therapy) and also at screening, 1 and 4 wk for IPSS, and 4 wk for BII. Statistical significance was interpreted only if the results of the preceding analysis were significant at the 0.05 level.

**Results:**

After 2 months of treatment the change from baseline to week 12 relative to “Tradamixina plus Seronea Repens” in total IPSS and Qol was statistically significant. Differences from baseline in BII were statistically significant for “Tradamixina plus Seronea Repens” above all differences in BII were also significant at 4 wk (LSmean ± SE: -0.8 ± 0.2). In the distribution of subjects over the PGI-I and CGI-I response categories were significant for”Tradamixina plus Seronea Repens” (PGI-I: p = 0.001; CGI-I). We also observed a decrease of total PSA.

**Conclusion:**

The daily treatment with a new compound “Tradamixina plus Serenoa Repens” for 2 months improved the male sexual function , it improved the bother symptoms which affect the patient’s quality of life , improved uroflowmetric parameters, and we also observed a decrease of serum PSA level.

## Background

Lower urinary tract symptoms (LUTS) are associated with great emotional costs [1] to individuals and substantial economic costs to society [2]. The prevalence and severity of LUTS increases with age [3], and the progressive growth of the aged population group has broadened the societal impact of LUTS. LUTS comprise storage symptoms (daytime urinary frequency, nocturia, urgency, urinary incontinence) voiding symptoms (slow stream, splitting or spraying, intermittency, hesitancy, straining, terminal dribble), and post micturition symptoms (sensation of incomplete emptying, post micturition dribble) [4] In EPIC, 62.5% of 7210 men in the five countries surveyed reported one or more LUTS; the prevalence of individual LUTS in men increased with age. A greater percentage of men reported storage symptoms (51.3%) vs. voiding (25.7%) or post micturition (16.9%) symptoms. Nocturia, defined by the ICS as waking one or more times to urinate during the night, was the most commonly reported symptom (48.6% of men); terminal dribble (14.2% of men) and sensation of incomplete emptying (13.5% of men) were the most commonly reported voiding and post micturition symptoms, respectively [5]. A large-scale multinational study revealed that 90%of men aged 50 to 80 suffer from potentially troublesome LUTS [3]. Questionnaire data from 1,271 men with LUTS indicated that many men have storage and voiding symptoms [6]. The same study demonstrated that voiding symptoms were the most common male LUTS, but that storage symptoms made up four of the five most bothersome LUTS. Although LUTS are also highly prevalent in women, their frequent comorbidity with prostatic disease in men adds complexity to the management of male LUTS [6]. Benign prostatic hyperplasia (BPH) is a pathologic process that contributes to, but is not the sole cause of, lower urinary tract symptoms (LUTS) in aging men. Despite intense research efforts in the past five decades to elucidate the underlying etiology of prostatic growth in older men, cause-and effect relationships have not been established. For example, androgens are a necessary but not a clearly causative aspect of BPH. Previously held notions that the clinical symptoms of BPH are due simply to a mass-related increase in urethral resistance are too simplistic. It is now clear that a significant portion of LUTS is due to age –related detrusor dysfunction. Bladder outlet obstruction itself may induce a variety of neural alteration in the bladder, which contributes to symptomatology. Moreover bothersome LUTS may be seen on men with polyuria, sleep disorders, and a variety of systemic medical conditions unrelated to the prostate- bladder unit. BPH is but one cause of the LUTS in aging men commonly, and probably incorrectly, referred to as prostatism. BPH is a classical age-related disease and present in 20% of men at the age of 40 years, with progression to 70% at the age of 60 years [7]. The clinical relevance of this disorder is underscored by the fact that up to 50% of elderly men develop lower urinary tract symptoms (LUTS) due to BPH/BPE, and that transurethral resection of the prostate remains one of the most frequent interventions in elderly men, with a lifetime risk for surgery of around 25–30% [7]. Histopathologically, BPH is characterized by an increased number of epithelial and stromal cells around the urethra with an excessive nodular growth localized to the points where ejaculatory ducts enter into the transitional or periurethral zones of the prostate. At the cellular level, alterations including basal cell hyperplasia (enlarged, hypertrophic basal cells), increased stromal mass (particularly the amount of smooth muscle cells), enhanced extracellular matrix deposition, reduced elastic tissue, more infiltrating lymphocytes around ducts, acinar hypertrophy and more luminal corpora amylacea and calcifications in the form of prostatic calculi [8]. Periurethral nodules in BPH compress the urethra and may cause urodynamic obstruction. Such an obstruction can lead to LUTS as well as secondary changes that may ultimately require surgical intervention, such as bladder hypertrophy, urinary tract infection development of post-void residual volume, upper urinary tract changes and urinary retention. The observed increase in cell number may be due to epithelial and stromal proliferation or to impaired programmed cell death leading to cellular accumulation. Androgens, estrogens, stroaml, epithelial interactions, growth factors, and neurotransmitters may play a role, either singly or in combination in the etiology of the hyperplastic process. The prostate receives innervations from the sympathetic and the parasympathetic nerve system. The sympathetic system (noradrenergic nerves) is responsible for expelling prostatic fluid into the urethra during ejaculation [9], and the parasympathetic system (cholinergic nerves) increases the rate of secretion [10]. Moreover, the neuronal system has been shown to regulate prostatic function and growth [11]. Neuronal systems with effects on the prostate include the alpha adrenergic [12], the beta adrenergic [13] the cholinergic [14], the enkephalinergic [15], the peptidergic [16] and the nitrinergic system [13].^.^Sympathetic signaling pathways are important in the pathophysiology of LUTS, as reviewed subsequently. In addition, there is increasing evidence that sympathetic pathways may be important in the pathogenesis of the hyperplastic growth process. Alpha blockade, in some model systems can induce apoptosis [17,18] .α –adrenergic pathways can also modulate the smooth muscle cell phenotype in the prostate[19]. All the components of the rennin-angiotensin system are present in prostatic tissue and may be active in BPH [20]. The alpha-1-adrenoreceptor is the prime determinant for urethral resistance causing outflow obstruction and LUTS [21]. Based on this observation, an important cornerstone of medical management of LUTS due to BPH/BPE is based on alpha-1-adrenergic-receptor (adrenoreceptor) blockade to reduce urethral resistance. This study seeks to evaluate the effect of a new natural compound “tradamixina “ made of Alga Ecklonia Bicyclis, Tribulus Terrestris and D-Glucosamine plus Serenoa Repens in order to improve lower urinary tract symptoms. Seven phlorotannins were isolated and characterized from an edible marine brown alga *Ecklonia Bicyclis*, along with three common sterol derivatives (fucosterol, ergosterol, and cholesterol) according to the comprehensive spectral analysis of MS and NMR data. Compounds 7-phloro eckoland ,6,6′-bieckoll in phlorotannin derivatives were obtained for the first time with their respective high yields. Any bioactive report of compound Fucodiphloroethol G was found nowhere up to date [22]. Ecklonia bicyclis has radical scavenger activity 10-100 times more powerful than any other polifenol terrestris plants, which have only 3-4 fenolic and rings that are commonly considered among the most effective antioxidant molecules. Common polyphenols are soluble in water also and have a relatively short half-life introduced into the body. All phlorotannins had antioxidant properties in vitro, especially, compounds 6,6′-bieckol which showed significant activities compared to the other phlorotannins [23]. In the Ecklonia bicyclis there are molecules that are able to reduce the inflammatory response, partially neutralizing the inflammatory damage caused by ROS and in part by slowing the gaming lipoxygenase and inhibiting the formation of prostaglandin E2, a powerful inflammatory mediator. *Jung Wk *[24] revealed that Ecklonia bicyclis inhibits LPS-induced NO and PGE_2_ production in a concentration-dependent manner and inhibits inducible iNOS and COX-2 in BV2 microglia without significant cytotoxicity. Ecklonia bicyclis treatment significantly reduced NF-kB translocation and DNA-binding in LPS-stimulated BV2 microglia. This effect was mediated through the inhibition of the degradation of the inhibitor kappaB and by inhibition of the mitogen-activated protein kinase (MAPK) phosphorylation, at least in part by inhibiting the generation of reactive oxygen species. This data also indicate that Ecklonia bicyclis extracts exert anti-inflammatory effects by suppressing proinflammatory cytokines. Collectively, these results suggest that Ecklonia bicyclis suppresses the induction of cytokines by LPS, as well as iNOS and COX-2 expression, by blocking NF-kappaB and MAPK activation. These findings provide mechanistic insights into the anti-inflammatory and neuroprotective actions of Ecklonia bicyclis in BV2 microglia [24]. *Won -Kyo Jung*[25] revealed that also only dieckol suppresses LPS-induced production of nitric oxide (NO) and prostaglandin E_2_ (PGE_2_) and expression of inducible nitric oxide synthase (iNOS) and cyclooxygenase-2 (COX-2) in a dose-dependent manner, without causing cytotoxicity. It also significantly reduced the generation of proinflammatory cytokines, such as interleukin (IL)-1β and tumor necrosis factor (TNF)-α. Moreover, dieckol significantly reduced LPS-induced nuclear factor κB (NF-κB) and p38 mitogen-activated protein kinases (MAPKs) activation, as well as reactive oxygen species (ROS) production. Taken together, the inhibition of LPS-induced NO and PGE_2_ production might be due to the suppression of NF-κB and p38 MAPK signal pathway and, at least in part, by inhibiting the generation of ROS. (25) *S.-K. Kim* revealed extracts reduced the concentrations of IL-4 and IL-5 by 66% and 84%, respectively, and resulted in a 73% reduction in the secretion of TNF-α . Ecklonia bicyclis extracts enhanced IFN-γ production, but not to a significant degree [26]. The protodioscin is a steroidal saponin, which is about 45% of the extract obtained from aerial parts of Tribulus Terrestris. Its particular steroidal structure has an androgen-mimetic action, binding and activating the receptor of testosterone. So this substance is able to increase the endogenous production of testosterone, dihydrotestosterone, a hormone luteinizing hormone (LH), dehydroepiandrosterone (DHEA) and dehydroepiandrosterone sulfate (DHEA-S). Because of these effects in experimental animals there is an increase in spermatogenesis and the frequency of matches. In the rabbit in particular it has been shown that the compound stimulates the release of nitric oxide (NO) by vascular endothelium of the corpora cavernosa thereby having a pro-erectile effect. The mechanism behind this effect appears to involve the pathway of steroid hormones. Although in humans protodioscin is used for the treatment of erectile dysfunction [27,28]. In a placebo-controlled study on a group of young volunteers serum levels of testosterone, androstenedione and luteinizing hormone were detected after administration of Tribulus Terrestris at doses of 10 and 20 mg / kg. After 4 weeks of treatment, these values were similar to those of untreated [29]. Biovis contains polymers of d-glucosamine and n-acetyl-d-glucosamine that act on both the non-adrenergic and non-colinergic system (NANC) and on the endothelial cell system as a strong nitric oxide synthetase (NOS) stimulator [30]. Serenoa Repens has been approved in France and Germany for treatment of BPH [31]. The mechanism of action of Serenoa Repens has been investigated in several in vitro or indirect in vivo studies and has not been definitively defined. The mechanism may include alteration of cholesterol metabolism, anti-oestrogenic, anti-androgenic (including 5a-reductase inhibitor activity), anti-inflammatory effects, and a decrease in available sex hormone binding globuline [32,34].

## Methods

An observational study was conducted from May 2011 to May 2012, at our Department of Urology. We enrolled 100 patients. Eligible men were ≥45 yrs. of age who had had LUTS/BPH for >6 mo at screening and with IPSS (The international Prostate symptom scores) ≥13 and maximum urinary flow rate (Qmax) ≥4 to ≤15 ml/s. Exclusion criteria were: drug assumption :α-blocker , Serenoa Repens , dutasteride, finasteride; hyper- and hypothyroidism, neurogenic syndrome (multiple sclerosis, multiple atrophy, Parkinson’s disease, tumors, stroke, disk disease, spinal cord disorders, polyneuropathy, uraemia), lower pelvic surgery (oncological pelvic surgery, lower urinary and genital tract surgery), prostate cancer. The compound “Tradamixina plus Serenoa Repens” (80 mg of Alga Ecklonia Bicyclis, 100 mg of Tribulus Terrestris and 100 mg of D-Glucosamine and N-Acetyl-D-Glucosamine plus 320 mg of Serenoa Repens) was administered daily for two months. At visit patients were evaluated by means of detailed medical urological history, clinical examination, laboratory investigations (total PSA), and instrumental examination like uroflowmetry. Efficacy measures included IPSS-International Prostate Symptom Scores (primary measure), BPH Impact Index (BII), and week 1 IPSS (mIPSS) questions beginning with ‘‘Since your last visit.’’ IPSS storage and voiding subscores, nocturia question (question 7), and IPSS Quality-of-Life (QoL) Index were also assessed. Measures were assessed at baseline and end point (12 wk or end of therapy) and also at screening, 1 and 4 wk for IPSS, and 4 wk for BII. The Patient and Clinician Global Impression of Improvement (PGI-I and CGI-I, respectively) instruments and the subject-rated Treatment Satisfaction Scale–BPH (TSS-BPH) [22], evaluated from 0% (greater) to 100% (lower) satisfaction, were administered at end point. Uroflowmetry was performed using standard calibrated devices at the screening, baseline, and end point visits. Valid Qmax measurements required prevoid total bladder volume (assessed by ultrasound) of ≥150 to ≤550 ml and voided volume (Vvoid) of ≥125 ml. Bladder capacity was calculated post hoc as the sum of Vvoid and postvoid residual (PVR) volume. Safety was evaluated based on subject-reported adverse events (AE), PVR, clinical laboratory parameters (total PSA). The primary efficacy objective was evaluating the change in total IPSS from baseline to end point. Efficacy was analysed in all subjects. At last continuous efficacy measures, uroflowmetry, and PVR were evaluated as a change from baseline to week 12/last-observation carried-forward end point. All other efficacy analyses (including all tradamixina results) were assessed at the 0.05 significance level without adjustment for multiplicity. A fixed-sequence testing procedure was implemented to control type I error in analyses of primary and key secondary outcomes for “Tradamixina plus Serenoa Repens” using the following pre-specified order: total IPSS at end point, total IPSS after 4 wk, BII at end point, mIPSS after 1 wk, and BII after 4 wk. Statistical significance was interpreted only if results of the preceding analysis were significant at the 0.05 level. Results were presented independent of the fixed sequence, as all end points tested under this procedure achieved statistical significance. All other efficacy analyses were assessed at the 0.05 significance level without adjustment for multiplicity. PGI-I- Patient Global Impression of Improvement- was analysed using the Cochran –Mantel-Haenszel test adjusted for baseline LUTS severity .Changes from baseline to end of therapy in Qmax, PVR, and clinical laboratory parameters were analysed using a ranked analysis of variance (ANOVA) with a term for treatment group. Treatment group differences for average urinary flow rate (Qave), Vvoid, and bladder capacity were performed as post hoc analyses.

## Results and discussion

Mean age was 64 yrs. of age (10.2% ±75 yr of age). At randomisation, IPSS was ≥20 in 30% of subjects, and Qmax was <10 ml/s in 54%. The change from baseline to week 12 relative to “Tradamixina plus seronea Repens” in total IPSS was statistically significant p = 0.001 (Table 1). Least squares mean (LSmean) plus or minus standard error (SE) differences in IPSS were significant for “Tradamixina plus Serenoa Repens” at 1 wk (mIPSS: -1.5 ± 0.5; p = 0.003 ) and 4 wk (-2.2 ± 0.6; p < 0.001 ). Changes in IPSS subscores and nocturia are shown in table 1. Differences from baseline in BII were statistically significant for “Tradamixina plus Seronea Repens” ( p = 0.003), above all differences in BII were also significant at 4 wk (LSmean ± SE: -0.8 ± 0.2;p < 0.001 ). For the IPSS QoL Index, significant improvements at 12 wk were reported ( p = 0.022).(Table 2). The TSSBPH overall satisfaction score at end point was significantly low (indicating higher satisfaction) ( p = 0.005).In the distribution of subjects over the PGI-I and CGI-I response categories were significant for “Tradamixina plus Seronea Repens” (PGI-I: p = 0.001; CGI-I: p = 0.004). More subjects and their clinicians perceived improvements in LUTS at end point . Improvements in Qmax were significantly great (p = 0.009) (Table 3). For PVR, mean reductions from were observed with “Tradamixina plus Serenoa Repens”, but were not statistically significant. We also observed a decrease of total PSA (Table 4). “Tradamixina plus Serenoa Repens” improved total IPSS score and PGI-I and CGI-I scores because the Ecklonia bicyclis with its anti-inflammatory action and antioxidant effects, suppress LPS-induced production of nitric oxide (NO) and prostaglandin E_2_ (PGE_2_) and expression of inducible nitric oxide synthase (iNOS) and cyclooxygenase-2 (COX-2) in a dose-dependent manner, without causing cytotoxicity. It also significantly reduced the generation of proinflammatory cytokines, such as interleukin (IL)-1β and tumor necrosis factor (TNF)-α. Moreover, dieckol significantly reduced LPS-induced nuclear factor κB (NF-κB) and p38 mitogen-activated protein kinases (MAPKs) activation, as well as reactive oxygen species (ROS) production [25]. It improved the bother symptoms. BPH is associated with changes of innervations, and biological mediator production and release in the central zone of the prostate [35]. In particular, there is a decrease of nerves of the enkephalinergic [36] and nitrinergic systems [37,38] both mediating smooth muscle cell relaxation [37]. Compared to normal tissue, nNOS expression has been observed to decrease in the transitional zone of BPH tissue. On the other hand, inducible NOS (iNOS), produced after stimulation by immune and inflammatory cytokines and free radicals, has been reported to increase selectively in the stroma of patients suffering from BPH [36]. This observation is probably due to increased proinflammatory conditions in BPH. The importance of the NOS system for the prostate stroma is further supported by experiments with constitutive active NOS dependent guanylylcyclases. cGMP analogues have been shown to activate the Proteinkinase G II and to inhibit proliferation of human smooth muscle cells in vitro [37]. Two enzymes, the neuronal (NOS-I) and the endothelial (NOS-III) isoforms, are Ca2_-dependent and constitutively expressed.The third enzyme is an inducible Ca2_-independent isoform (NOS-II), expressed after stimulation with *Escherichia coli* lipopolysaccharide (LPS) and/or different cytokines, such as interferon-γ (IFNγ), interleukin-1, or tumor necrosis factor- NOS-II induction occurs at the transcriptional level and is mediated by the early activation of some nuclear transcriptional factors, including NFkB [38]. A large body of experimental evidence suggests that physiological levels of NO, similar to those produced by the basal activity of NOS-I or NOS-III, prevent induction of NOS-II mRNA expression through the suppression of NFkB activation [39,40]. As a consequence, NOS-II gene expression takes place after LPS/cytokine stimulation, provided that the NOS-I- or NOS-III-generated NO is reduced below a threshold value in a short time [41]. A recent report [42,43] shows that NOS-II inducers (*e.g.* LPS and IFNγ) consistently elicit a rapid inactivation of NOS-I by tyrosine phosphorylation, an event leading to a decrease of basal NO levels. A recent study [44] reports that inhibition of NOS-I can be achieved via activation of cytosolic phospholipase A2 (cPLA2), a large molecular mass member of the family of PLA2 enzymes. The activities of NOS-I and cPLA2 are both regulated by increases in the intracellular concentration of free Ca2 ([Ca2]*i*). Not surprisingly, enhancing the [Ca2]*i* caused a parallel increase in both activities and accumulation of respective products, NO and arachidonic acid (AA). Inducible nitric oxide synthase (iNOS) is expressed in a variety of cell types, in particular in inflammatory cells, in response to diverse pro-inflammatory stimuli. This process requires critical levels of arachidonic acid (AA), generated by constitutive phospholipase A2 (PLA2), promoting tyrosine kinase-dependent phosphorylation, and inhibition, of constitutive NOS. Lowering basal NO levels is indeed critical for the activation of NF-κB, and thus for the expression of genes (e.g. iNOS) regulated by this transcription factor. It is interesting to note that NO and AA, two small lipid soluble molecules, rapidly cross the plasma membrane thereby allowing the triggering of the above responses in distal cells. That is, constitutive NO might inhibit NF-κB activity in the same cells (e.g. astrocytes) in which it is generated, as well as in other cells that do not express constitutive NOS (e.g. microglia). NO from cells unable to respond to pro-inflammatory stimuli (e.g. neurons) will also contribute to these effects. Along the same line, AA released by pro-inflammatory molecules in specific cell types (e.g. astrocytes) might suppress constitutive NOS activity in the same cells as well as in other cells (e.g. neurons). Thus, AA produced at the very early stages of the inflammatory response is a likely critical signal switching the regulation of the “NO tone” from physiological (i.e. mediated by constitutive NOS) to pathological (i.e. mediated by iNOS). This second phase of the inflammatory response is often accompanied by the onset of deleterious effects in the tissue in which a critical role is played by iNOS-derived NO (directly or indirectly, i.e. via formation of peroxynitrite) as well as by products of the AA cascade. In summary, the relative amounts of NO and AA, released by their constitutive enzymes, produce autocrine and paracrine effects regulating the onset of an inflammatory response in which, in addition to other factors, NO and AA are extensively released by their inducible enzymes [45]. Biovis contains polymers of d-glucosamine and n-acetyl-d-glucosamine that act both on the non-adrenergic and non-colinergic system (NANC) and on the endothelial cell system as a strong nitric oxide synthetase (NOS) stimulator [46]. This explains why there is an improvement of Qave and Qmax. In fact while α-blocker drugs facilitated the opening of the bladder neck thanks to the presence of alpha receptors, Tradamixina improved the NOS action on its receptor, so for the reasons above also improved LUTS. Serenoa Repens also has anti-inflammatory effects. As described above, α1-adrenoceptor antagonists are commonly used in the treatment of men with voiding symptoms (urinary obstruction, pollakiuria and urinary incontinence) secondary to BPH. Goepel *et. Al.* have shown that Serenoa Repens might have α1-adrenoceptor inhibitory properties. Serenoa Repens significantly affects pharmacological receptors, such as the α1-adrenoceptor and the muscarinic receptor in the lower urinary tract, to relieve the irritative and obstructive symptoms of dysuria due to BPH and LUTS [34]. In addition to traditionally used medications, like α1-adrenoceptor antagonists, antimuscarinics, 5α-reductase inhibitors, and phytotherapy, several new therapeutic agents, such as selective β3-adrenoceptor agonists, are potentially useful for treating LUTS suggestive of BPH, particularly for storage symptoms secondary to outflow obstruction [47]. Thus, the effects of SPE on these receptors in the lower urinary tract might be pharmacologically relevant. To date, more than 11 placebo-controlled trials and 4 active-controlled trials with SPE in men with BPH have been conducted. Patient numbers were usually limited and the evaluation periods were relatively short, so it would be difficult to evaluate the effect of SPE and ascertain the efficacy of SPE in BPH patients. However, some placebo-controlled studies and comparisons to α1-blockers have recently been conducted with relatively long-term treatments and sufficient numbers of patients [48-50]. BPH causes dysuria and residual urine *via* a mechanical stoppage due to hypertrophy of prostatic tissue and *via* a functional stoppage caused by α1-adrenoceptor hypertonia of prostatic smooth muscle. Previous studies have demonstrated that Serenoa Repens had a number of pharmacological effects: 1) an antiandrogenic effect — inhibition of 5α-reductase I and II and inhibition of binding of dihydrotestosterone (DHT) to the cytosolic androgen receptors, 2) an anti-inflammatory effect, 3) an anti-proliferative effect, and 4) significant binding of pharmacological receptors existing in the lower urinary tract. In BPH there is a decreased ratio between androgen and estrogen, and tribulus terrestris by increasing total testosterone serum level restores the ratio.

**Table 1:** International prostate symptom score (IPSS) total,storage and voiding subscores and nocturia question (IPSS question 7).

*IPSS total:*	
Change from baseline ,LS mean ±SE	-6,3±0,5 p= 0.001

***Storage subscore ^1^***	

Change from baseline ,LS mean ±SE	-2,2±0,2 p= 0.055

***Voiding subscore^2^***	

Change from baseline ,LS mean ±SE	-4,1± 0.3 p< 0,001

***Nocturia question^3^***	

Change from baseline ,LS mean ±SE	-0,5± 0.13 p= 0,080

1) IPSS question: 2+4+7

2) IPSS question: 1+3+5+6

3) IPSS question:7

**Table 2:** International Prostate Symptom Score Quality of Life Index, Treatment Satisfaction scale, and Patient or Clinician Global Impression of Improvement Scores at 12 wks. compared to baseline

*IPSS total Qol index*	
Change from baseline ,LS mean ±SE	-1,3±0,1

***TSS-BPH overall***	

mean±SD	26,9±17,7

***PGI-I no.***	

Very much better	58
Much better	35
A little better	5
No change	2
A little worse	0
Much worse	0
Very much worse	0

***CGI-I no.***	

Very much better	41
Much better	30
A little better	15
No change	14
A little worse	0
Much worse	0
Very much worse	0

**Table 3:** Uroflowmetry and postvoid residual volume

*Qmax ml/s:*	
Baseline	9.9±3.6
Mean change	2,4±5.5

***Q ^ave^ ml/s***	

Baseline	5,9±2,1
Mean change	1,6±3,2

***V ^void^ ml***	

Baseline	257.7±94.3
Mean change	8.2±101.5

***Bladder capacity*** **(*ml*)**	

Baseline	310±109.4
Mean change	3,5±113.8

***PVR* (*ml*)**	

Baseline	53,3±50,4
Mean change	-4,6±47,0

Qmax = maximum flow rate; Qave = average flow rate; Vvoid = voided volume; PVR = postvoid residual volume.

**Table 4:** 

Total PSA	
Baseline	3.6±2,4
Mean change	1,1±0,2

## Conclusion

The daily treatment with a new compound “Tradamixina” (100 mg of Alga Ecklonia Bicyclis, 80 mg of Tribulus Terrestris and 80 mg of D-Glucosamine and N-Acetyl-D-Glucosamine) plus 320 mg Serenoa Repens for two months improved the male sexual function. It improved the bother symptoms which affect the patient’s quality of life, improved uroflowmetric parameters, and we observed a decrease of serum PSA level. These effects are due to its antioxidant, anti-aging action, and the bother symptoms due to its anti-inflammatory action. Infact it neutralizes the action of ROS, LPS, COX2, NFkβ, probably also reducing the concentrations of TNF-α, MMP-1. The decrease of PSA is due to the anti-inflammatory action. This result can be the basis for future research.

## List of abbreviations

AA: Arachidonic acid; AE: Adverse events; BII: BPH Impact Index; BPH: Benign prostatic hyperplasia; CGI-I: The Clinician Global Impression of Improvement; COX-2: Cyclooxygenase-2; cPLA2: Cytosolic phospholipase A2; DHEA: Dehydroepiandrosterone; DHEA-S: Dehydroepiandrosterone sulfate; IL-1β: Interleukin; iNOS: Inducible nitric oxide synthase; IPSS: International Prostate Symptom; IPSS: International Prostate Symptom; LH: Hormone luteinizing hormone; LUTS: Lower urinary tract symptoms; MAPKs: Mitogen-activated protein kinases; MMP-1: Matrix metalloproteinase-1; NANC: Non-adrenergic and non-colinergic system; NF-κB: Nuclear factor κB; NO: Nitric oxide; NOS: Nitric oxide synthetase; NOS-I: Neuronal Nitric oxide synthetase isoforms I; NOS-III: Endothelial Nitric oxide synthetase isoforms III; PGE_2_: Prostaglandin E_2_; PGI-I: Patient Global Impression of Improvement; PGI-I: The Patient and Clinician Global Impression of Improvement; PVR: Postvoid residual; Qave: Urinary flow rate; QoL: Quality-of-Life; ROS: Reactive oxygen species; TNF-α: Tumor necrosis factor; TSS-BPH: Treatment Satisfaction Scale–BPH; Vvoid: Voided volume

## Competing interests

The authors declare that they have no competing interests.

## Authors’ contributions

FI, DP: conception and design, interpretation of data, given final approval of the version to be published; EI, AR, GR: acquisition of data, drafting the manuscript, given final approval of the version to be published; BA: critical revision, interpretation of data, given final approval of the version to be published.
